# The profile of the key pro-inflammatory cytokines in the serum of patients with CD and their association with the disease severity and activity

**DOI:** 10.1186/s12876-022-02562-w

**Published:** 2022-11-21

**Authors:** Ahmed Al Qteishat, Kiril Kirov, Dmitry Bokov

**Affiliations:** 1 Department of Biological Sciences and Chemistry, University of Nizwa, PC 616, Birkat Al-Mouz, 33, Nizwa, Sultanate of Oman; 2 Research Institute, Medical University Pleven, Sv. Kliment Ohridski Str., 1, Pleven, 5800 Bulgaria; 3 Institute of Pharmacy, Sechenov First Moscow State Medical University, Trubetskaya Str., 8/2, Moscow, 119991 Russian Federation; 4 Laboratory of Food Chemistry, Federal Research Center of Nutrition, Biotechnology and Food Safety, Moscow, Russian Federation

**Keywords:** Crohn’s disease, Pathogenesis, Cytokines, Immune system, Blood

## Abstract

**Background:**

The epidemiology of Crohn’s disease (CD) has changed over the past decades, demonstrating a trend toward increased prevalence in developing countries, while in developed countries, its incidence has stabilized. The study aimed to examine the profile of the key pro-inflammatory cytokines in the serum of patients with CD and establish their association with the severity and activity of the disease.

**Methods:**

A total of 61 patients (29 women (47.5%), 32 men (52.5%) aged from 18 to 40 years (mean age (30.42 ± 2.51) years) with the verified diagnosis of CD in the active phase were examined. The control group consisted of 30 healthy people of corresponding age.

**Results:**

CD is characterized by a reliable increase of pro-inflammatory cytokines in blood compared to healthy people: tumor necrosis factor-α (TNF-α) – by 4.45 times (137.46 ± 9.72 vs. 30.88 ± 2.08 pg/ml in healthy people, p < 0,001), interleukin-1α (IL-1α) – by 5.08 times (51.55 ± 4.36 vs. 10.14 ± 0.93 pg/ml, *p* < 0.001), interleukin-6 (IL-6) – by 2.16 times (20.03 ± 1.81 vs. 9.27 ± 0.52 pg/ml, *p* < 0.001), interleukin-8 (IL-8) – by 2.04 times (25.74 ± 2.05 vs. 12.62 ± 1.16 pg/ml, *p* < 0.001), and interferon-γ (IFN-γ) – by 5.30 times (208.63 ± 14.29 vs. 39.35 ± 2.40 pg/ml, *p* < 0.001). The authors have established direct correlations between the Crohn's disease activity index and blood content of TNF-α (*r* = 0.84, *p* < 0.013), INF-γ (*r* = 0.61, *p* < 0.028); between TNF-α and INF-γ content (*r* = 0.67, *p* < 0.023), IL-1α (*r* = 0.49, *p* < 0.042), IL-6 (*r* = 0.40, *p* < 0.045), and IL-8 (*r* = 0.51, *p* < 0.033); INF-γ and IL-1α (*r* = 0.53, *p* < 0.040), IL-6 (*r* = 0.37, *p* < 0.039), IL-8 (*r* = 0.44, *p* < 0.040).

**Conclusions:**

Patients with CD were found to have multiple cytokines (TNF-α, IL-1α, IL-6, IL-8, and IFN-γ,). The content of cytokines correlated positively with the CD activity index.

## Introduction

CD, like ulcerative colitis (UC), is an inflammatory bowel disease (IBD) with a prevalence ranging from 0.1–58 cases per 100,000 people, depending on the region [1]. More than 2 million people in North America and 3.2 million people in Europe suffer from this disease [2]. CD is most common among people aged 20 to 30 years [3, 4]. The relevance of CD is not only because its prevalence is increasing annually but also since full-fledged treatment requires high direct and indirect costs throughout the lives of patients, not to mention the psychological and emotional distress of these people and the deterioration of their life’s quality [5, 6].

CD affects a very specific area of the gastrointestinal tract (GIT), the ileocecum [7–9]. It can occur elsewhere only after surgery changing the primary site of fecal impaction [10]. In particular, it can involve the oral cavity. The causative agent is the *Mycobacterium avium subsp. paratuberculosis* (MAP) [11, 12].

However, according to modern data, the basis of the pathogenesis of CD is the loss of immunological tolerance in the gastrointestinal tract to a set of MAP antigens, as well as to related polymorphic variants [11–13]. At the same time, the induction of immune tolerance to MAP occurs when the acquired immunity is clearly underdeveloped [13]. In the case of insufficiency or absence of acquired immunity in the neonatal period, an infection caused by MAP changes the immune memory; therefore, upon repeated contact with the MAP antigen, immune tolerance is lost [12, 14]. As a result, the immune system responds with a pro-inflammatory reaction, while a whole set of cytotoxic cytokines are produced, which target the areas of epithelial attachment and antigen-processing dendritic cells and macrophages [13, 15]. Despite the fact that the epithelium of the gastrointestinal tract has high regenerative capabilities, as a result of frequent immune attacks on the intestinal mucosa, it is damaged, especially in areas of significant fecal impaction. At the same time, as a result of local changes in redox potential, commensal microorganisms reach disease-causing potential and change the composition of the bacterial microflora of the gastrointestinal tract. For the debut of the disease, repeated exposure to the complex of MAP antigens is necessary, which explains the presence of a latent period between infection and the next disease, while active replication of MAP is not necessary for the induction of CD [11, 15].

Given the fact that repeated contact with the MAP antigen causes a pro-inflammatory reaction with the production of a number of cytokines, in recent years more and more attention has been paid to the role of various cytokines in the pathogenesis of CD, including tumor necrosis factor-α (TNF-α), interleukin-1 (IL-1), IL-2, IL-6, IL-8, IL-12, IL-18, and interferon-γ (IFN-γ) [16–18]. Among pro-inflammatory cytokines, TNF-α has the greatest significance in the development of CD. Its excess in the body is associated with a number of the following biological processes: activation of T- and B-lymphocytes, neutrophils with the induction of IL-2, INF-γ; activation of macrophages with the induction of IL-2, IL-6 synthesis; activation of free radical synthesis; synthesis of acute-phase pro-inflammatory proteins in the liver (seromucoid, C-reactive protein, α1-antitrypsin, and others); development of inflammatory reactions (leukocytosis, sepsis, fever, weight loss); development of endotoxemia; increase in vascular wall permeability with subsequent migration of leukocytes to the inflammation focus; stimulation of adhesion molecules expression on endotheliocytes and leukocytes; inhibition of apoptosis of inflammatory cells [19, 20]. In CD, the concentration of IL-1, IL-2, IL-6, IL-8, and TNF-α sharply increases, while the concentration of anti-inflammatory cytokines (IL-4, IL-10, IL-11, and others) decreases [21].

### Objectives

The significant importance of cytokines in the pathogenesis of CD determines the necessity to perform detailed studies of their content depending on the disease course, stage, and pathogenesis. Given the features of the cytokine profile of a particular patient, their examination as predictors of the disease severity and markers of inflammatory process activity would allow developing individual therapy tactics, providing the predictive treatment of CD.

*The aim of the study* was to investigate the profile of the main pro-inflammatory cytokines in the serum of patients with CD and establish their association with the disease severity and activity.

## Materials and methods

A study enrolled 61 patients (29 women (47.5%), 32 men (52.5%) aged from 18 to 40 years (mean age (30.42 ± 2.51) years) diagnosed with CD in an active phase. The control group consisted of 30 healthy people of the corresponding age. The study was conducted from 2015 to 2019.

Patients who met the following requirements were included in the study: the diagnosis of CD in the active phase (confirmed by the results of colonoscopy and histology); age from 18 to 40 years; a voluntary consent form signed by the patient to participate in the study.

Verification of CD was performed in accordance with 2018 Recommendations of the American College of Gastroenterology [8], and the European Crohn’s and Colitis Organization [22], based on the results of colonoscopy and histological examination of biopsy specimens of the affected colon area.

All patients included in the study underwent a detailed interview with an examination of complaints, medical and life history, physical examination, general clinical, biochemical, and instrumental examinations.

Disease activity was determined by calculating the CD activity index (CDAI), which is based on an assessment of clinical disease manifestations: frequency of mushy stool, abdominal pain, general condition, other symptoms (including extraintestinal and intestinal complications), abdominal muscle tension, administration of antidiarrheal drugs, hematocrit, body weight. According to CDAI grading, clinical remission is indicated by a value of fewer than 150 points, low activity (mild disease severity) by 150–300 points, moderate activity (moderate disease severity) by 301–450 points, and high activity (severe disease severity) by more than 450 points.

The following laboratory tests were performed: general clinical blood and urinalysis, coprological examination, fecal occult blood test, determination of blood glucose, total protein, albumin and globulin, urea, creatinine, C-reactive protein, total, direct and indirect bilirubin, hepatic transaminases activity, and coagulogram. Blood sampling for the biochemical study was performed from the ulnar vein on an empty stomach in the morning.

The blood content of cytokines (TNF-α, INF-γ, IL-1α, IL-6, IL-8) was determined by enzyme immunoassay (ELISA) using ELISA Kit test systems (Diaclone SAS, France) on Stat Fax 3030 Plus analyzer (USA). Blood cells were incubated in the presence of lipopolysaccharide (as a mitogen), phytohemagglutinin, and concavalin-A, as well as in a culture medium (RPMI-1640) for 24–48 h at 37 °C in a 5% CO_2_ atmosphere. The samples (400 g) were then centrifuged for 10 min, and the supernatant was used for further testing.

All patients underwent obligatory colonoscopy for endoscopic verification of the diagnosis. Each colonoscopy was accompanied by a biopsy for histological verification of CD diagnosis. Besides, every patient underwent an ultrasound examination of the abdominal and pelvic organs, electrocardiography, and chest X-ray examination.

The results were statistically processed using methods of variance statistics, such as Mann–Whitney U-test. The correlation analysis was performed using the Spearman method. Microsoft XP Excel (2013) and Statistical Package for the Social Sciences (SPSS) 17.0 were applied for statistical data processing.

### Ethics approval

The research was conducted according to the ethical standards established in the 1964 Declaration of Helsinki and its later amendments or comparable ethical standards. The study protocol was approved by University of Nizwa. Written informed consent was obtained from patients to participate in the study.

### Consent to participate

Informed consent was obtained from all individual participants included in the study.

## Results

The mean age of CD diagnosis in examined patients was (27.75 ± 3.62) years.

The study of the features of CD clinical course showed that the most typical symptoms for the included patients were asthenia-vegetative being observed in 61 people(100.0%), abdominal pain in 55 people (90.2%), flatulence in 46 people (75.4%), diarrhea/frequent stool in 40 people (65.6%), an admixture of mucus and/or blood in stool in 32 people (52.5%), weight loss in 39 people (63.9%), increased body temperature in 37 people (60.7%). Besides, 30 patients (49.2%) with CD had extraintestinal manifestations, among which joint lesions were in 13 (21.3%) patients, skin lesions in 10 patients (16.4%), gallstone disease in 8 patients (13.1%), urolithiasis in 7 patients (11.5%), and eye lesions in 7 patients (11.5%). It should be noted that among 30 patients (49.2%), extraintestinal symptoms with involvement of several organs and organ systems were recorded in 16 patients (53.3%, Table 1).

**Table 1:** Distribution of clinical symptoms and disease activity (according to CDAI) in patients with Crohn’s disease (*n* = 61)

Characteristics	No. of patients	%
*Main clinical symptoms*		
astheno-vegetative	61	100.0
abdominal pain	55	90.2
flatulence	46	75.4
diarrhea/frequent stools	40	65.6
mucus and/or blood in stool	32	52.5
weight loss	39	63.9
temperature rise	37	60.7
*Nonintestinal manifestations*		
joint lesions	13	21.3
skin lesions	10	16.4
cholelithiasis	8	13.1
eye diseases	7	11.5
*Disease activity*		
low	18	29.5
moderate	37	60.7
high	6	9.8

When analyzing the CDAI values, 18 patients (29.5%) corresponded to low disease activity, 37 patients (60.7%) had moderate activity, and high activity of the disease was noted in 6 (9.8%) patients. The mean CDAI value in patients was (346.90 ± 25.37) points, which corresponds to a moderate degree of disease severity. Besides, CDAI was higher in persons with a combined involvement of the large and small intestine lesions than those with terminal ileitis or isolated involvement of the large intestine.

Compared to healthy people, the study of the pro-inflammatory cytokines content in the blood of CD patients showed an increase in the following proteins (Table 2): TNF-α increased 4.45-fold (137.46 ± 9.72 vs. 30.88 ± 2.08 pg/ml in healthy people, *p* < 0.001), IL-1α – 5.08-fold (51.55 ± 4.36 vs. 10.14 ± 0.93 pg/ml, *p* < 0.001), IL-6 – 2.16-fold (20.03 ± 1.81 vs. 9.27 ± 0.52 pg/ml, *p* < 0.001), IL-8 – 2.04-fold (25.74 ± 2.05 vs. 12.62 ± 1.16 pg/ml, *p* < 0.001), and INF-γ – 5.30-fold (208.63 ± 14.29 vs. 39.35 ± 2.40 pg/ml, *p* < 0.001).

**Table 2:** Serum levels of pro-inflammatory cytokines in patients with Crohn’s disease, (M ± SD)

Indicator	Healthy people (*n* = 30)	Patients with Crohn’s disease (*n* = 61)
TNF-α, pg/ml	30.88 ± 2.08	137.46 ± 9.72^a^
IL-1α, pg/ml	10.14 ± 0.93	51.55 ± 4.36^a^
IL-6, pg/ml	9.27 ± 0.52	20.03 ± 1.81^a^
IL-8, pg/ml	12.62 ± 1.16	25.74 ± 2.05^a^
IFN-γ, pg/ml	39.35 ± 2.40	208.63 ± 14.29^a^

^a^ The difference is statistically significant compared to healthy people (*p* < 0.005)

It has been established that the blood content of the pro-inflammatory cytokines increased with higher disease activity (CDAI). In particular, TNF-α content in the blood of patients with low cytokines activity was 3.34 times higher than that in healthy people (*p* < 0.001), with moderate activity – by 4.41 times (*p* < 0.001), with high activity – by 5.70 times (*p* < 0.001). At that, the content of this cytokine in persons with moderate disease activity was 1.32 times (*p* < 0.005) higher than in persons with low activity, 1.30 times (*p* < 0.005) higher in persons with moderate disease activity, 1.71 times (*p* < 0.001) higher in persons with low activity of the disease (Fig. 1).

**Fig. 1:** TNF-α content (pg/ml) in blood serum of patients with Crohn’s disease as a function of the disease activity stage. Note. The «▬» sign in chart blocks denotes the mean value of indicators

A similar trend was observed for the IFN-γ content in the blood. Thus, this indicator was 4.24 times (*p* < 0.001) higher than in persons with low disease activity than in healthy people, 5.08 times higher (*p* < 0.001), in those with moderate activity, and 5.99 times higher in patients with highly active disease course (*p* < 0.001). At that, IFN-γ content in people with moderate activity was 1.28 times (*p* < 0.005) higher compared to patients with low disease activity, and those with high activity had 1.20 times (*p* < 0.005) higher content compared to moderate activity and 1.54 times (*p* < 0.005) higher compared to low activity (Fig. 2).

**Fig. 2:** The INF-γ content (pg/ml) in blood serum of patients with Crohn’s disease as a function of the disease activity stage. Note. The «▬» sign in chart blocks denotes the mean value of indicators

IL-1α content was 3.65 times (*p* < 0.001) higher in those with low disease activity, 5.00 times (*p* < 0.001) with moderate activity, and 6.14 times (*p* < 0.001) with high activity, respectively. In those with moderate CD activity, this cytokine content was 1.37 times (*p* < 0.001) higher than by low activity higher than in low activity, and in patients with high activity – 1.27 times (*p* < 0.001) higher than with moderate activity and 1.73 times (*p* < 0.001) higher than with low activity (Fig. 3).

**Fig. 3:** The IL-1α content (pg/ml) in blood serum of patients with Crohn’s disease as a function of the disease activity stage. Note. The «▬» sign in chart blocks denotes the mean value of indicators

Compared to healthy people, the IL-6 content in the blood of patients with low disease activity was 1.96 times higher (*p* < 0.001), with moderate activity – 2.15 times higher (*p* < 0.001), and with high activity – 2.55 times (*p* < 0.001) (Fig. 4). The content of IL-8 was 1.68 (*p* < 0.005), 1.96 (*p* < 0.005), and 2.39 times higher (*p* < 0.001) higher, respectively (Fig. 5). Patients with high CD activity demonstrated 1.31 times higher (*p* < 0.005) IL-6 blood content compared to patients with low disease activity and 1.43 times higher (*p* < 0.005) IL-8 content compared to patients with low disease activity, respectively.

**Fig. 4:** The IL-6 (pg/ml) in blood serum of patients with Crohn’s disease as a function of the disease activity stage. Note. The «▬» sign in chart blocks denotes the mean value of indicators

**Fig. 5:** The IL-8 content (pg/ml) in blood serum of patients with Crohn’s disease as a function of the disease activity stage. Note. The «▬» sign in chart blocks denotes the mean value of indicators

The following correlations have been established: between the CD activity index and the content of TNF-α (*r* = 0.84, *p* < 0.013), INF-γ (*r* = 0.61, *p* < 0.028); between TNF-α and INF-γ content (*r* = 0.67, *p* < 0.023), IL-1α (*r* = 0.49, *p* < 0.042), IL-6 (*r* = 0.40, *p* < 0.045), and IL-8 (*r* = 0.51, *p* < 0.033); INF-γ and IL-1α (*r* = 0.53, *p* < 0.040), IL-6 (*r* = 0.37, *p* < 0.039), IL-8 (*r* = 0.44, *p* < 0.040); IL-1α and IL-6 (*r* = 0.55, *p* < 0.045), IL-8 (*r* = 0.36, *p* < 0.038); IL-6 and IL-8 (*r* = 0.60, *p* < 0.020).

## Discussion

According to the study results, the term of CD diagnosis in examined patients was quite late and amounted to years, which coincides with the data of other studies [23, 24]. The patients included in the study demonstrated typical clinic features of CD with a predominance of asthenic-vegetative and abdominal pain syndromes, stool disorders, weight loss, and others. However, rather a large part of patients had extraintestinal lesions. The most common of them was the damage of joints as arthropathies and skin lesions as erythema nodosum (Table 1). The development of skin lesions in CD patients is associated with the TRAF3IP2 gene and HLA-B*27, HLA-B*58, and HLADRB1*0103 antigens [25]. In general, the occurrence of extraintestinal lesions during CD is associated with the ability of the intestinal mucosa to induce an immune response in extraintestinal sites. That is due to the presence of common epitopes in intestinal microorganisms, particularly in the synovial membrane. An adaptive immune response is stimulated due to the bacteria move through the intestinal barrier, which had a high permeability [1, 26]. Hence, the results of this study regarding the main clinical manifestations of CD and extraintestinal lesions coincide with the available literature findings [7, 26, 27].

According to the results of this study, the CD was characterized by a significant increase of such pro-inflammatory cytokines as TNF-α, INF-γ, IL-1α, IL-6, and IL-8 in the blood content, whose values varied within a fairly wide range (Table 2). Such high content is attributed to the development of an active inflammatory process in the intestine and a systemic reaction of the body. It should be noted that in patients with CD the growth was in TNF-α content and IFN-γ, which is comparable to the results of studies by other scientists. This increase in TNF-α and IFN-γ content in the examined patients confirms their leading role in the cascade of immune-inflammatory reactions during CD. In particular, being synthesized by macrophages, monocytes, T- and B-lymphocytes, detritus cells, neutrophils, keratinocytes, and endotheliocytes, TNF-α has a wide range of biological effects. Besides, it activates the proliferation of fibroblasts and lymphocytes; increases the expression of adhesion molecules (both cellular and vascular) necessary for lymphocyte migration to the inflammatory zone; stimulates the synthesis of leukotrienes, prostaglandins, matrix metalloproteinases, nitrogen monoxide; decreases body weight [17, 28]. At CD, TNF-α directs circulating inflammatory cells to its focus, resulting in edema formation. This cytokine also initiates coagulation processes and participates in granuloma formation [17].

This study shows that another cytokine playing a crucial pathogenetic role in developing CD is INF-γ, also called immune interferon. This cytokine is produced by T-lymphocytes (CD4 + and CD8 +) and NK cells. IFN-γ is involved in the stimulation of Tx0 to Tx1, maintenance of Tx1/Tx2 balance, regulation of cellular and humoral immune response (it enhances cellular immunity development while inhibiting its humoral link), mediates the relationship between lymphocytes and macrophages, perform antiviral and anti-tumor activity [17, 27, 28].

The patients with CD included in the study were characterized by a significant increase in IL-1α content compared to healthy people), but no correlation between this cytokine content in blood and disease severity (Best activity index) has been established. The increase of IL-1α in serum during CD can be explained by the fact that this cytokine is one of the main inflammation mediators but is less specific concerning the disease under study. The IL-1α is necessary to activate T-cells during their interaction with antigen being the main mediator of short-distance activity (it remains inside the cell or can have a membrane form and may appear only in insignificant amounts in the extracellular space) [17].

The increase of IL-6 and IL-8 content in the blood was less significant (Table 2). Besides, no correlation between the content of the indicated cytokines and the disease severity (Best’s activity index) was found, which may indicate their secondary role in the CD pathogenesis.

### Limitations of the study

Patients with at least one of the following criteria were excluded from the study: CD in remission stage; age less than 18 years and older than 40 years; other inflammatory diseases of GIT; acute somatic pathology; other chronic somatic pathology in acute or sub/decompensation stage; infectious diseases; cancer pathology of any localization; mental diseases; pregnancy, lactation.

## Conclusions

Patients with CD were found to have multiple cytokines (TNF-α, IL-1α, IL-6, IL-8, and IFN-γ,). Cytokine levels correlated positively with the CD activity index.

### Prospect for further research

The prospect for further research is to study the quantitative and qualitative composition of the intestinal microbiome in patients with CD, as well as the possibility of using probiotic drugs in the complex treatment of this disease.

## Data Availability

The datasets generated during and/or analysed during the current study are not publicly available due to privacy and ethical restrictions but are available from the corresponding author on reasonable request.

## Abbreviations

CD: Crohn’s disease
UC: Ulcerative colitis
IBD: Inflammatory bowel disease

## References

[1] Roda G, Ng SC, Kotze PG, Argollo M, Panaccione R, Spinelli A (2020). Crohn’s disease Nat Rev Dis Primers.

[2] Ananthakrishnan AN, Kaplan GG, Ng SC (2020). Changing global epidemiology of inflammatory bowel diseases-sustaining healthcare delivery into the 21st century. Clin Gastroenterol Hepatol.

[3] Ng SC, Shi HY, Hamidi N, Underwood FE, Tang W, Benchimol EI (2018). Worldwide incidence and prevalence of inflammatory bowel disease in the 21st century: a systematic review of population-based studies. Lancet.

[4] King D, Reulen RC, Thomas T, Chandan JS, Thayakaran R, Subramanian A (2020). Changing patterns in the epidemiology and outcomes of inflammatory bowel disease in the United Kingdom: 2000–2018. Aliment Pharmacol Ther.

[5] De Jong MJ, Boonen A, van der Meulen-de Jong AE, Romberg-Camps MJ, van Bodegraven AA, Mahmmod N (2020). Cost-effectiveness of telemedicine-directed specialized vs standard care for patients with inflammatory bowel diseases in a randomized trial. Clin Gastroenterol Hepatol.

[6] Lichtenstein GR, Shahabi A, Seabury SA, Lakdawalla DN, Espinosa OD, Green S (2020). Lifetime economic burden of Crohn’s disease and ulcerative colitis by age at diagnosis. Clin Gastroenterol Hepatol.

[7] Pimentel AM, Rocha R, Santana GO (2019). Crohn’s disease of esophagus, stomach and duodenum. World J Gastrointest Pharmacol Ther.

[8] Lichtenstein GR, Loftus EV, Isaacs KL, Regueiro MD, Gerson LB, Sands BE (2018). ACG clinical guideline: management of Crohn’s disease in adults. Am J Gastroenterol.

[9] Rohr M, Narasimhulu CA, Sharma D, Doomra M, Riad A, Naser S (2018). Inflammatory diseases of the gut. J Med Food.

[10] Bala N, Gupta N, Singh N, Nandan G, Sachdeva M. A rare case presentation of Warty dyskeratoma involving multiple adjoining follicles. ETDHR-V9. 2022;9:163–6.

[11] Pierce ES (2018). Could Mycobacterium avium subspecies paratuberculosis cause Crohn’s disease, ulcerative colitis and colorectal cancer?. Infect Agent.

[12] Safonov V, Ermakov V, Danilova V, Yakimenko V (2021). Relationship between blood superoxide dismutase activity and zinc, copper, glutathione and metallothioneines concentrations in calves. Biomath.

[13] Monif GRG (2015). The Hruska postulate of Crohn’s disease. Med Hypotheses.

[14] Ventsova I, Safonov V (2021). Biochemical criteria for the development mechanisms of various reproduction disorders in dairy cows. Biodivers J Biolog Divers.

[15] Monif GRG (2021). The Crohn’s disease: The Infectious Disease Incorporated’s Perspective. Gastrointest Discord.

[16] Bevivino G, Monteleone G (2018). Advances in understanding the role of cytokines in inflammatory bowel disease. Expert Rev Gastroenterol Hepatol.

[17] Friedrich M, Pohin M, Powrie F (2019). Cytokine networks in the pathophysiology of inflammatory bowel disease. Immunity.

[18] Marafini I, Sedda S, Dinallo V, Monteleone G (2019). Inflammatory cytokines: from discoveries to therapies in IBD. Expert Opin Biol Ther.

[19] Ostrikov A, Ospanov A, Vasilenko V, Muslimov NZ, Timurbekova AK, Jumabekova GB (2019). Melt flow of biopolymer through the cavities of an extruder die: mathematical modelling. Math Biosci Eng.

[20] Ostrikov A, Ospanov A, Shevtsov A, Vasilenko V, Timurbekova A (2021). An empirical-mathematical modelling approach to explore the drying kinetics of cereals under variable heat supply using the stitched method. Acta Agric Scand Section B: Soil Plant Sci.

[21] Bertani L, Baglietto L, Antonioli L, Fornai M, Tapete G, Albano E (2020). Assessment of serum cytokines predicts clinical and endoscopic outcomes to vedolizumab in ulcerative colitis patients. Br J Clin Pharmacol.

[22] Gomollón F, Dignass A, Annese V, Tilg H, Van Assche G, Lindsay JO (2017). 3rd European evidence-based consensus on the diagnosis and management of Crohn’s disease 2016: Part 1: diagnosis and medical management. J Crohn’s Colitis.

[23] Biancone L, Zuzzi S, Ranieri M, Petruzziello C, Calabrese E, Onali S (2012). Fistulizing pattern in Crohn’s disease and pancolitis in ulcerative colitis are independent risk factors for cancer: a single-center cohort study. J Crohn’s Colitis.

[24] Moon JM, Kang EA, Han K, Hong SW, Soh H, Park S (2020). Trends and risk factors of elderly-onset Crohn’s disease: a nationwide cohort study. World J Gastroenterol.

[25] Chavez-Álvarez S, Gómez-Flores M, Ocampo-Candiani J (2016). Cutaneous manifestations in inflammatory bowel disease. Gac Med Mex.

[26] Vavricka SR, Schoepfer A, Scharl M, Lakatos PL, Navarini A, Rogler G (2015). Extraintestinal manifestations of inflammatory bowel disease. Inflamm Bowel Dis.

[27] Nemeth ZH, Bogdanovski DA, Barratt-Stopper P, Paglinco SR, Antonioli L, Rolandelli RH (2017). Crohn’s disease and ulcerative colitis show unique cytokine profiles. Cureus.

[28] Roggenbuck D, Reinhold D, Baumgart DC, Schierack P, Conrad K, Laass MW (2016). Autoimmunity in Crohn’s disease-a putative stratification factor of the clinical phenotype. Adv Clin Chem.

